The article "Abnormalities of the Default Mode Network Functional Connectivity in Patients with Insomnia Disorder" was published in 2022. Journal: Contrast Media Mol Imaging.

# Abnormalities of the Default Mode Network Functional Connectivity in Patients with Insomnia Disorder

**DOI:** 10.1155/2022/9197858

**Published:** 2022-08-27

**Authors:** Guangyuan Xia, Yongxue Hu, Fangxian Chai, Yiming Wang, Xingde Liu

**Affiliations:** ^1^Department of Psychology, The Affiliated Hospital of Guizhou Medical University, Guiyang, Guizhou Province 550004, China; ^2^Guizhou Medical University, Guiyang 550004, China; ^3^Department of Cardiology, The Second Affiliated Hospital of Guizhou University of Traditional Chinese Medicine, Guiyang 550004, China

## Abstract

**Objective:**

This paper aimed to probe changes in the default mode network (DMN) functional connectivity (DMNFC) of the brain of patients with insomnia disorder (ID) under the resting state.

**Methods:**

A total of 67 patients with ID and 67 graphically matched healthy controls were selected. Then, their general information was collected, followed by a psychological scale valuation. Resting state functional magnetic resonance imaging (rs-fMRI) scanning was conducted. Subsequently, collected statistics were processed, bilateral precuneus and medial superior frontal gyrus were defined as regions of interest (ROI), and the difference in intensity between these two groups was compared.

**Results:**

Compared with the healthy control group, the patients in the ID group were observed with abnormalities of DMNFC. Specifically, a significant increase in the functional connectivity (FC) could be observed between the left medial superior frontal gyrus and left central anterior gyrus, the left medial superior frontal gyrus and anterior cingulate gyrus, the right medial superior frontal gyrus and left central anterior gyrus, the left anterior cuneiform and left central anterior/posterior gyrus, the left anterior cuneiform and left superior occipital gyrus, as well as the right anterior cuneiform and left central posterior gyrus. However, the FC between the left anterior cuneiform and the right middle frontal gyrus was weakened, as well as between the left anterior cuneiform and the right angle gyrus and between the right precuneus and the left inferior temporal gyrus.

**Conclusion:**

ID patients may suffer changes in FC. The decline of FC in DMN may be one of the underlying causes of ID; the enhancement of FC between DMN and the visual-spatial attention network may play a key role in the mechanisms of impaired brain functional networks of ID.

## 1. Introduction

Insomnia disorder (ID), one of the most common sleep disorders [1, 2], affects 10% of adults. ID is defined as a lasting disorder in falling asleep, time of sleep, the persistence of sleep, and quality of sleep [3], which can result in or is accompanied by daytime dysfunctions [4]. Besides, ID induces adverse outcomes like the decline in recognition function and disorder in emotional regulation and then affects the health of human beings.

The article "Abnormalities of the Default Mode Network Functional Connectivity in Patients with Insomnia Disorder" was published in 2022. Journal: Contrast Media Mol Imaging.

The temporal correlation between the activities of the brain functional network and each encephalic region is analyzed by functional connectivity (FC) analysis methods based on resting state functional magnetic resonance imaging (rs-fMRI), further reflecting the intensification of the correlation among different encephalic regions [5].

Currently, most of the rs-fMRI studies focus on unveiling the population differences of subjects, but this approach has certain drawbacks when it comes to classifying or predicting individuals. Moreover, some inconsistent conclusions have been drawn from some research studies on insomnia in the default mode network (DMN). Significant reductions in FC were found between ventromedial prefrontal cortex (vmPFC) and the right medial temporal lobe and between vmPFC and the left medial parietal cortex. While some other studies have also revealed that patients with insomnia have higher connectivity between nodes in the posterior cingulate or hippocampus and the DMN [6]. To realize individualized clinical evaluation, we compared the statistics of a single patient with those of a group. In predicting the model of early stages of insomnia, the default network's precuneus and medial superior frontal gyrus account for a large portion of the final outcome. This paper aimed to further study the pathogenesis of insomnia based on the FC of the seed points of the precuneus and medial superior frontal gyrus, find the effective biomarker indicators that could diagnose and evaluate insomnia, and provide the physiological mechanism of neurologic cases of insomnia with new foundations.

## 2. Materials and Methods

### 2.1. Materials

In the ID group, 67 cases were confirmed to be ID in the Department of Psychology, Affiliated Hospital of Guizhou Medical University, from July 2019 to January 2020. All insomniacs met the criteria of the ID group after diagnosis by two senior doctors with the professional titles. The inclusion criteria of the ID group were as follows. The enrolled patients needed to (1) meet the criteria set by the ICSD-3 ID diagnosis, i.e., patients suffered from insomnia thrice a week, lasting for more than three months; (2) patients aged 20–60 years old; (3) right hander (confirmed by the Edinburgh handedness questionnaire [7]); and (4) without taking benzodiazepines and nonbenzodiazepines before entering the group. The exclusion criteria of subjects were as follows. Patients (1) suffered from other major mental disorders, (2) contraindications for MRI, (3) degenerative diseases of the nervous system or major physical diseases, and (4) were pregnant and lactating.

The article "Abnormalities of the Default Mode Network Functional Connectivity in Patients with Insomnia Disorder" was published in 2022. Journal: Contrast Media Mol Imaging.

As for the healthy control group, 65 healthy volunteers were recruited through advertisements (matched with the ID group on gender, age, and educational level). The criteria set for the control group were as follows. The chosen patients aged (1) from 20 to 60 years old, (2) did not meet the diagnostic criteria of any DSM-IV psychiatric disorder, (3) slept well and on time one week before the experiment, and (4) were right-handed without mental disorder among first-degree relatives. The exclusion criteria were as follows. Patients suffered from (1) brain or physical disease that affected brain functions, (2) contraindications for MRI, and (3) were in pregnancy or lactation.

All subjects in this study signed informed consent and volunteered to participate in this research. The research procedure was approved by the Research Ethics Committee of the Affiliated Hospital of Guizhou Medical University (2020477).

### 2.2. Psychological Scale Valuation

Physicians in the Department of Psychiatry with senior titles assessed the quality of sleep and depressive state of subjects using the Pittsburgh Sleep Quality Index (PSQI), insomnia severity index (ISI), Epworth Sleepiness Score (ESS), and Hamilton Depression Scale (HAMD-17).

### 2.3. Magnetic Resonance Imaging Scan

All the brain image data in this research were collected by professional and technical personnel in the imaging department located in the 3.0 T Magnetic Resonance Room, Department of Imaging, and Affiliated Hospital of Guizhou Medical University. Data were collected using Philips Achieva 3.0 T magnetic resonance scanner made in The Netherlands and Sense-XL-Torso 8-channel cranial coil. To be specific, the subjects were asked to lie on their backs, stay awake, keep eupnea, fix their heads in comfortable positions, and limit the movement of their heads and limbs to the utmost. Also, they were asked to keep their eyes closed, move passively, and avoid any thinking activity. All scanning operations of MRI were completed by the same doctor in one imaging department. The doctor first scanned the subjects on the conventional sequence like T1WI, T2WI, and FLAIR to exclude those suffering from intracranial organic lesions, then scanned the rest of the subjects on rs-fMRI and 3D-T1WI sequence. Rs-fMRI adopted the Echo Planar Imaging (EPI) scanning sequence, and the specific parameters were as followed: Time of Repetition (TR) = 2000 ms, Time of Echo (TE) = 30 ms, Field of Vision (FOV) = 200 × 220 mm, Flip Angle = 90°, Pixel = 3.4 × 3.4 mm^2^, Layer Thickness = 3.4 mm, Number of Layers = 35, Time of *S* = 6 min 46 sec. Parameters scanned by the 3D-T1WI sequence were shown as follows: TR = 12 ms, TE = 5.9 ms, FOV = 250 × 250 mm, Pixel = 0.6 × 0.6 mm^2^, Layer Thickness = 1 mm, Number of Layers = 257, Time of Scanning = 7 min 45 sec.

The article "Abnormalities of the Default Mode Network Functional Connectivity in Patients with Insomnia Disorder" was published in 2022. Journal: Contrast Media Mol Imaging.

### 2.4. Preprocessing of Magnetic Resonance Imaging Data

The image data were preprocessed through SPM12 and rs-fMRI statistic processing box CONN18b. Specifically, researchers eliminated the first five time points, rectification of the time layer, and rectification of head movement (excluding the statistics of subjects whose head movement was larger than 3 mm or 3°). Also, the statistics by spatial standardized collection were eliminated according to the standard brain template provided by the Montreal Neurological Institute and the liner drift and low pass filtering (0.01 ≤ *f* ≤ 0.08 Hz). Additionally, the standardized data were processed smoothly with a half-height, full-width Gaussian kernel to the increase signal-to-noise ratio.

### 2.5. Functional Connectivity Analysis

Through the method of correlation of seed point, the collected statistics between an individual subject and the subjects in a group were compared, and the weight diagram of the ID prediction model was then obtained. The top 5% of encephalic regions (i.e., precuneus and medial superior frontal gyrus) with the highest weights were defined as seed points. Moreover, the method of time correlation was adopted to compute the FC value of the bilateral medial superior frontal gyrus, precuneus, and the whole brain. After FC analysis, age, gender, and education were regarded as concomitant variables, and the analysis results were corrected on the basis of the cluster-level FEW or FDR. *P* < 0.05 indicated the statistical significance of the final outcome of the computation.

### 2.6. Statistical Processing

SPSS22.0 software was utilized to process the collected data statistically and study the population informatics of the subjects. The data normality were first tested. In terms of age, years of education, PSQI, ISI, ESS, and HAMD-17 score, a two-sample *T* test was used to determine the differences between the two groups. The chi-square test was adopted to analyze the differences in the two groups on gender formation, marriage, and exercise (Exercise standards: brisk walking, jogging, cycling, rope skipping, mountain climbing, and swimming more than three times a week, each lasting more than 25 minutes, and the exercise intensity should be controlled below 140 beats per minute). *P* < 0.05 suggested that the analyzed data were statistically significant. FC analysis was performed after the processing of magnetic resonance data; precuneus and medial superior frontal gyrus were defined as seed points [8]. Moreover, the method of time correlation was utilized to compute the FC value of bilateral medial superior frontal gyrus, precuneus, and the whole brain. The obtained results were corrected on the basis of the cluster-level FEW or FDR, and *P* < 0.05 was considered as the judgment criterion of statistical significance.

The article "Abnormalities of the Default Mode Network Functional Connectivity in Patients with Insomnia Disorder" was published in 2022. Journal: Contrast Media Mol Imaging.

## 3. Results

### 3.1. Comparison of the ID and Healthy Control Groups

This research enrolled 67 insomniacs (average age: 33.73 ± 10.20 years; years of education: 15.21 ± 3.27; 44 females and 23 males) and 65 healthy controls in the control group (average age: 32.78 ± 11.50 years; years of education: 16.62 ± 2.84; 38 females and 23 males). There were no distinct differences in age, gender, and years of education between the two groups (*P* > 0.05).

### 3.2. Score Comparisons of ID and Healthy Control Groups

Compared with the healthy control group, the ID group had significantly higher PSQI and ISI (*P* > 0.05).

### 3.3. Comparisons of FC Values between the ID and Healthy Control Groups

After comparing the DMNs of the two groups, an obvious enhancement of FC values was observed among the left medial superior frontal gyrus, left anterior central gyrus, and anterior cingulate gyrus of the ID group (Figure 1), between the right medial superior frontal gyrus and left anterior central gyrus (Figure 2), and among the left precuneus, left central/posterior gyrus, and left suprapoccipital gyrus; while the FC values among the left precuneus, right middle frontal gyrus, and right angular gyrus were decreased (Figure 3). Additionally, the FC values between the right precuneus and the left posterior central gyrus were increased, whereas those between the right precuneus and the left inferior temporal gyrus were decreased (Figure 4). The intensification and weakening of the specific FC in different encephalic regions are shown in Tables 3 and 4.

The functional connectivity among the left medial superior frontal gyrus, left anterior central gyrus, and anterior cingulate gyrus was enhanced in chronic insomnia patients. Results were corrected by cluster level FWE, *P* < 0.05.

The functional connectivity was enhanced between the right medial superior frontal gyrus and the left anterior central gyrus in ID patients. Results were corrected by cluster level FWE, *P* < 0.05.

The functional connectivity among the left precuneus, left posterior central gyrus, and left suprapoccipital gyrus was increased, while the functional connectivity among the left precuneus, right middle frontal gyrus, and right angular gyrus was decreased. Results were corrected by cluster level FWE, *P* < 0.05.

The article "Abnormalities of the Default Mode Network Functional Connectivity in Patients with Insomnia Disorder" was published in 2022. Journal: Contrast Media Mol Imaging.

The functional connectivity between the right precuneus and the left posterior central gyrus was increased, while the functional connectivity between the right precuneus and the left inferior temporal gyrus was decreased. Results were corrected by cluster level FWE, *P* < 0.05.

### 3.4. Correlation Analysis of Brain Regions with the Abnormal Functional Connectivity Values, PSQI, and ISI in the ID Group

On the basis of the correlation analysis on the ID group, when the left medial superior frontal gyrus was considered as the seed point, the FC values of the anterior cingulate gyrus (*r* = 0.451, *P* = 0.001, *r* = 0.338, *p* ≤ 0.001) and left anterior central gyrus (*r* = 0.324, *P* = 0.016; *R* = 0.402, *p* = 0.001) were positively correlated with the PSQI and ISI scores. When the right precuneus was set as the seed point, the FC value of the left posterior central gyrus (*r* = 0.333, *P* = 0.013; *R* = 0.418, *p* = 0.008) had a positive correlation with PSQI score, while that of the left inferior temporal gyrus exhibited a negative correlation (*r* = −0.662, *P* = 0.001; *R* = 0.402, *p* ≤ 0.001). When the left precuneus served as the seed point, the FC value of the left superior occipital gyrus was positively correlated with PSQI and ISI scores (*r* = 0.438, *P* = 0.001; *R* = 0.495, *p* = 0.011).

## 4. Discussion

Under the resting state, some parts of the human brain, like the posterior cingulate cortex (PCC), precuneus, and medial prefrontal cortex, show high cerebral blood flow and CO_2_ exhaustion [9] and exhibit continuously high levels of activation. While under the task state, signals in these parts are decreased and restrained. Currently, it is believed that DMN predominantly consists of the ventromedial prefrontal cortex, dorsomedial prefrontal cortex, PCC, precuneus, and transverse parietal cortex [10]. Some basic cognition activities that the brain executes under the minimally conscious state rely on the default network, so the DMN contributes to the maintenance of awareness, the enhancement of episodic memory, the monitoring and reflecting of the surroundings, and the regulation of emotions [11]. The DMN can compare the differences in the cognition functions that encephalic regions perform, which is valuable in studying mental diseases. However, studies on the default network system under the resting state remain limited. Past studies have shown that the occurrence of ID is closely related to DMN. Marques et al. [12] proposed that the rs-fMRI environment might form an environmental simulator to simulate the situation that typical ID faces at night. Procedures without mission requirements promote cognition activities within ID, thereby producing lasting negative cognition, like deep thinking and worries. Regen et al. [13] stated that the posterior cingulate and hippocampus shared big connectivity with nodes of the DMN. Nie et al. [14] discovered that the FC of patients with ID between the medial prefrontal cortex and the right medial temporal lobe decreased significantly, and such phenomenon also appeared between the left medial temporal lobe and the left subparietal cortex. Zhou et al. [15] observed that the encephalic regions of patients suffering from ID were significantly increased in the central part of DMN. A recent study conducted by Dong et al. [16] revealed that the task-activated brain network may stay alert even if the patient was in the resting state, and this finding was similar to the brain mode facing outside stimulus under task mode.

The article "Abnormalities of the Default Mode Network Functional Connectivity in Patients with Insomnia Disorder" was published in 2022. Journal: Contrast Media Mol Imaging.

One rs-fMRI research has reported that wide changes happen when patients with ID are in the resting state [17]. To be specific, the FC among the frontal lobe, occipital lobe, and anterior cingulate is decreased, whereas the FC between the limbic system and anterior cingulate is intensified. In the resting state, the major role that DMN plays is to help patients stay awake. The above research believes that the weakening of DMN functions may be related to the neurophysiological changes of ID. However, in this paper, we drew a different conclusion. We discovered that the FC between the medial superior frontal gyrus and anterior cingulate was intensified, which may be the result of patients' adaptation to the changes in the inner environment when facing the chronic course of the disease and long-term insomnia. Our conclusion is similar to that of Wang et al. [18].

Functionally, DMN can be categorized into pre-DMN centered on the medial prefrontal lobe and rear-DMN centered on the precuneus and angular gyrus [19]. Pre-DMN is concerned with self-referential psychological activities and shares close bonds with the anterior cingulate. As for post-DMN, it is closely related to the hippocampus and involved in the memory of previous experiences [20]. The functional balance between pre- and post-DMN matters to the normal cognition, emotion regulation, and sleep of patients. Some studies discovered that when healthy controls enter deep sleep from rapid eye movement sleep, the activity of pre-DMN drops, whereas that of post-DMN is enhanced [12]. Dong et al. [16] reported that compared with the healthy control group, the subjects of the ID group may face decreased FC in pre- and post-DMN. The research by Dong et al. suggested that the imbalance of pre- and post-DMN may be one of the reasons why patients with ID suffer from poor sleep quality. Our results also support the above standpoint, and we discovered that the FC among the left precuneus, right middle frontal gyrus, and right angular gyrus was decreased, as well as the right precuneus and left temporal gyrus. The above outcomes suggest changes in FC in pre- and post-DMN networks. Some other researchers have pointed out that patients suffering from ID may experience functional changes in multiple networks, and among these networks, DMN plays an intermediary role [13]. All in all, DMN may be the potential cause of insomnia.

The article "Abnormalities of the Default Mode Network Functional Connectivity in Patients with Insomnia Disorder" was published in 2022. Journal: Contrast Media Mol Imaging.

Additionally, in this study, compared with that of the healthy control group, the FC of the ID group between DMN and visuospatial network was intensified. Specifically, an obvious enhancement in FC could be observed between the left medial superior frontal gyrus and left anterior central gyrus, the right medial superior frontal gyrus and left anterior central gyrus, the left precuneus and left anterior central gyrus, as well as the left precuneus and gyri occipitals superiores. The brain's visual spatial attention network in the hippocampus can be categorized into ventral and dorsal attention networks. These two networks are major constituent parts of the attention networks [21]. Previous neuroimaging studies reported that regional disordered spontaneous nervous activities can be detected in the encephalic regions of the attention network of ID sufferers and sleep despoilers [22]. The hyperarousal of ventral and dorsal attention networks may be the core inducement of the inability of patients with ID to activate or sustain sleep [23, 24]. Damages in these two visual pathways may disturb the processing and visual properties of the object and stress the role these two attention networks play in sleep-related attention bias behavior, which may lead to patient's inability to activate or sustain sleep. Thus, the hyperarousal of the visual space network function may be an important part of the cause of ID.

However, this research is limited by the small sample size. Patients in this research cannot form a large enough sample to support further experiments. In the future, the number of subjects will be enlarged for further experiments.

## 5. Conclusion

On the basis of rs-fMRI statistics, we have analyzed the DMNFC in patients with insomnia by the FC method. Moreover, the analysis outcomes reveal that the functional changes in and between DMNs can help us to understand the potential mechanisms of the impaired brain functional networks of insomnia.

## Figures and Tables

**Figure 1:** Functional connectivity analysis based on the region of interest.

**Figure 2:** Functional connectivity analysis based on the region of interest.

The article "Abnormalities of the Default Mode Network Functional Connectivity in Patients with Insomnia Disorder" was published in 2022. Journal: Contrast Media Mol Imaging.

**Figure 3:** Functional connectivity analysis based on the region of interest.

**Figure 4:** Functional connectivity analysis based on the region of interest.

**Table 1:** Comparisons of the ID and the control groups ($\tilde{\chi }$ *±* *S*).

Items	Healthy control group	ID group	*P*
Number of cases	65	67	—
Age (years)	32.8 ± 11.5	33.7 ± 10.2	0.583
Gender	38F/27M	44 F/23M	0.087
Years of education	16.6 ± 2.8	15.2 ± 3.3	0.437
Marriage	36Y/29N	40Y/27N	0.694
Attendance of exercise	42Y/23N	38Y/29N	0.187
Age of morbidity	—	29.4 ± 10.7	—
Frequency of morbidity	—	1.5 ± 0.7	—
Duration of disease (month)	—	38.5 ± 50.1	—

F: female; M: male; Y: yes; N: no.

**Table 2:** Scores of sleep-related scale between the ID and the control groups ($\tilde{\chi }$ ± *S*).

	Healthy control group	ID group	*t*	*P*
*PSQI*				
Sleep quality	0.06 ± 0.25	2.52 ± 0.634	19.99	≤0.001^*∗*^
Sleep latency	0.19 ± 0.40	2.59 ± 0.825	14.44	≤0.001^*∗*^
Sleep duration	0.35 ± 0.48	2.52 ± 0.74	13.49	≤0.001^*∗*^
Sleep efficiency	1.78 ± 1.43	3.00 ± 0.12	4.61	≤0.001^*∗*^
Sleep disturbances	0.35 ± 0.49	1.52±-0.63	8.00	≤0.001^*∗*^
Sleep medication	0.06 ± 0.25	1.17 ± 1.13	5.29	≤0.001^*∗*^
Daytime dysfunction	0.26 ± 0.45	1.24 ± 0.87	5.55	≤0.001^*∗*^
Global score	6.7 ± 1.8	15.9 ± 2.3	17.82	≤0.001^*∗*^
ISI	3.6 ± 2.2	18.5 ± 4.0	23.35	≤0.001^*∗*^
*ESS*	1.9 ± 1.8	1.7 ± 1.8	0.17	0.893
HAMD-17	8.5 ± 4.8	11.5 ± 3.3	2.69	0.670

^*∗*^: In comparison of the control group with the ID group, *P* *<* 0.05 indicates that the difference between the two groups were statistically significant.

**Table 3:** Intensified encephalic regions between the ID group and the healthy control group.

Encephalic regions	*MNI coordinates*			Voxel (mm^3^)	Peak *t* value
	*x*	*y*	*z*		
Between the left medial superior frontal gyrus and the left anterior central gyrus	−30	−15	+51	383	5.36
Between the left medial superior frontal gyrus and the anterior cingulate gyrus	−06	+24	+36	219	5.08
Between the right medial superior frontal gyrus and the left anterior central gyrus	−48	−06	+48	229	4.66
Between the left precuneus and the left central/posterior gyrus	−54	−18	+54	701	4.79
Between the left precuneus and the left supraoccipital gyrus	−21	−69	+30	208	4.33
Between the right precuneus and the left posterior central gyrus	−60	−21	+48	492	5.17

**Table 4:** Weakening encephalic regions of the ID and healthy control groups.

Encephalic regions	*MNI coordinates*			Voxel (mm^3^)	Peak t value
	*x*	*y*	*Z*		
Between the left precuneus and the right angular gyrus	+54	−51	+45	131	−3.64
Between the left precuneus and the right middle frontal gyrus	+42	+33	+42	143	−4.15
Between the precuneus and the left inferior temporal gyrus	−51	−12	−42	171	−4.18

MNI: Montreal Neurological Institute.

The article "Abnormalities of the Default Mode Network Functional Connectivity in Patients with Insomnia Disorder" was published in 2022. Journal: Contrast Media Mol Imaging.

## Data Availability

The data used to support the findings of this study are available from the corresponding author upon request.
